# ADA-COVID: Adversarial Deep Domain Adaptation-Based Diagnosis of COVID-19 from Lung CT Scans Using Triplet Embeddings

**DOI:** 10.1155/2022/2564022

**Published:** 2022-02-08

**Authors:** Mehrad Aria, Esmaeil Nourani, Amin Golzari Oskouei

**Affiliations:** ^1^Faculty of Information Technology and Computer Engineering, Azarbaijan Shahid Madani University, Tabriz, Iran; ^2^Department of Computer Engineering, Faculty of Electrical and Computer Engineering, University of Tabriz, Tabriz, Iran

## Abstract

Rapid diagnosis of COVID-19 with high reliability is essential in the early stages. To this end, recent research often uses medical imaging combined with machine vision methods to diagnose COVID-19. However, the scarcity of medical images and the inherent differences in existing datasets that arise from different medical imaging tools, methods, and specialists may affect the generalization of machine learning-based methods. Also, most of these methods are trained and tested on the same dataset, reducing the generalizability and causing low reliability of the obtained model in real-world applications. This paper introduces an adversarial deep domain adaptation-based approach for diagnosing COVID-19 from lung CT scan images, termed ADA-COVID. Domain adaptation-based training process receives multiple datasets with different input domains to generate domain-invariant representations for medical images. Also, due to the excessive structural similarity of medical images compared to other image data in machine vision tasks, we use the triplet loss function to generate similar representations for samples of the same class (infected cases). The performance of ADA-COVID is evaluated and compared with other state-of-the-art COVID-19 diagnosis algorithms. The obtained results indicate that ADA-COVID achieves classification improvements of at least 3%, 20%, 20%, and 11% in accuracy, precision, recall, and F_1_ score, respectively, compared to the best results of competitors, even without directly training on the same data. The implementation source code of the ADA-COVID is publicly available at https://github.com/MehradAria/ADA-COVID.

## 1. Introduction

Nearly 268 million people worldwide officially have been infected with the COVID-19, and more than 5.2 million death tolls until November 2021 [1] as of epidemic declaration in March 2020 signify the rapid diagnosis of the COVID-19 with high reliability in the early stages, not only to save human lives but also to reduce the social and economic burden on the communities involved. Although the RT-PCR (real-time polymerase chain reaction) test is the standard reference for confirming COVID-19, some studies show that this laborious method cannot diagnose the disease in the early stages [2–5], and some studies report a high false-negative rate [6].

One standard way to identify morphological patterns of lung lesions associated with COVID-19 is to use chest scan images. There are two common techniques for scanning the chest: X-rays and computer tomography (CT). Detection of COVID-19 from chest images by a radiologist is time-consuming, and the accuracy of COVID-19 diagnosis depends strongly on the radiologist's opinion [7, 8]. Also, manually checking every image might not be feasible in emergency cases. Recently, deep learning-based methods [9, 10] have been applied to help the medical community diagnose COVID-19 quickly, accurately, and automatically.

Using CT images to diagnose COVID-19 has recently drawn researchers' interest due to some key ideas that they possess: more accurate images of bones, organs, blood vessels, and soft tissues. Using these images, radiologists can better identify internal structures in more detail and evaluate their texture, density, size, and shape. Chest images obtained by CT scan usually provide much more accurate images of the patient's condition than X-rays. Therefore, in recent works based on deep learning, CT scan images are used more than plain radiographs [11–14].

Deep learning-based methods usually require large datasets to achieve better results and overcome overfitting [15]. In the accurate detection of COVID-19 using chest images, the lack of comprehensive, high-quality datasets is a fundamental problem in this research area. The COVID CT dataset was first introduced in [16] and has been used in recent works [11–13]. The next SARS-CoV-2 CT scan dataset [17] contains 2,482 CT scan images collected from hospitals in São Paulo, Brazil. Another large dataset includes 7495 positive corona samples and 944 negative ones [18]. The mentioned datasets are the largest and most common datasets used in this field, while researchers also use other small public datasets [19–21].

It is observed that obtained evaluation results on test samples belonging to the same dataset used for training are significantly better than other datasets [22]. In other words, model performance is artificially good when the train and test sets belong to the same dataset. At the same time, model performance is dramatically reduced when the trained model is evaluated on another dataset. Numerous studies demonstrate that the most recent approaches in the literature are unreliable [23, 24]. For example, two well-known studies [10, 25] in this field show a performance close to random classification facing unseen data (i.e., datasets on which the model has not been trained). For example, the classification accuracy in research [22] decreases from 98.5% on the test set to 59.12% on unseen datasets. The structural and inherent differences in the images from the available datasets, which arise from different tools and medical imaging methods, are the cause of this issue. Upon closer inspection, we found that most of the proposed methods for detecting and classifying COVID-19 are trained and tested on a set of images from the same dataset. Using a single dataset during network training reduces the model generalization. One of the fundamental problems of deep learning is shortcut learning [26]. Decision rules that perform well on typical benchmarks but fail to transfer to more complex testing situations, such as real-world scenarios, are examples of shortcuts [26].

This paper proposes an adversarial deep domain adaptation-based approach for diagnosing COVID-19 from lung CT scan images, termed ADA-COVID. In ADA-COVID, two datasets with different input domains are used in the network training process. The goal is to generate similar representations for images belonging to two different domains. This model can perform the correct classification regardless of the specific features of each input distribution. In other words, the generated representations are domain invariant, and overall better representations are generated. Also, due to the excessive structural similarity of medical images compared to other image data in machine vision, we use the triplet loss function for the training model. Using this loss function, similar (dissimilar) representations are generated for samples of the same class (different classes) in the embedded space.

The contributions of this work are twofold:

1. The effect of structural and intrinsic differences in images obtained from different medical imaging tools and methods is minimized as a result of the introduced domain adaptation-based approach for CT images.
2. A custom deep model is designed based on this approach to make corona case detection more reliable. Therefore, the generalization of the ADA-COVID for other new datasets and in the real-world application is high.

The performance of the ADA-COVID method is evaluated on two standard datasets, and extensive experiments are performed to examine the effectiveness of each solution proposed. The results show that our approach achieves higher performance than the existing competitors.

The rest of the paper is organized as follows.  Section 2 gives a brief review of the related work; in Section 3, the proposed ADA-COVID is described in detail. In Section 4, the experimental results are presented. In Section 5, the conclusions and possible future works are discussed.

## 2. Related Work

With the prevalence of COVID-19, various methods were introduced to diagnose COVID-19 [14, 27–29]. These methods can be classified into three general categories: (1) methods that have developed customized network architectures specifically for COVID-19 detection, such as COVID-Net [10], COVID CT-Net [30], and CVR-Net [31], (2) methods that use pretrained networks and transfer learning to detect COVID-19, such as COVID-ResNet [32], CoroNet [33], COVID-CAPS [25], and convolutional CapsNet [34], and (3) very few studies employed handcrafted feature extraction approaches and conventional classifiers. In the following, we review each of these categories.

### 2.1. Methods Based on Customized Network Architectures

COVID-Net [10] is one of the earliest methods based on convolutional neural networks designed to detect COVID-19 using X-ray images. CVR-Net (Coronavirus Recognition Network) [31] is a customized model with convolutional layers trained and tested on a combination of CT and X-ray images. In CVR-Net, an average accuracy of 78% was reported for the CT image dataset. Further improvements were added to COVID-Net to improve its representational ability for one specific image modality and to make the network computationally more efficient [35]. CovidCTNet [36] is a set of open-source algorithms used to differentiate COVID-19 from community-acquired pneumonia (CAP) and other lung diseases. The aim of designing this model is to work with heterogeneous and small sample sizes independent of CT imaging hardware. In [13], an AUTOENCODER-based architecture was used to simultaneously segment and classify CT images. Their proposed architecture consists of an encoder and three decoders; these decoders are used for image reconstruction, image segmentation, and classification, respectively. COVID CT-Net [30] is an attentional CNN, which can focus on the infected areas of the chest. All of the introduced approaches in this category propose a customized architecture for detecting infected cases without utilizing any well-established pretrained networks.

### 2.2. Methods Based on Pretrained Models

In contrast to the first group, methods based on pretrained models have recently gained more attention, where standard pretrained CNN models are used to detect COVID-19 [37] based on CT images. In [38], convolutional networks and transfer learning have been used to classify the samples into three categories: COVID-19, bacterial pneumonia, and normal. This study aims to evaluate the performance of standard CNN models such as VGG19 [39], MobileNet v2 [40], Inception [41], Xception [42], and InceptionResNetV2 [41], which have been proposed in recent years. In [43], to detect COVID-19, transfer learning with fine-tuning has been used and evaluated their proposed method on four popular CNN architectures: ResNet18 [44], ResNet50 [44], SqueezeNet [45], and DenseNet-121 [46]. They prepared a dataset of around 5000 X-ray images for COVID-19 detection. Brunese et al. [47] used transfer learning on a pretrained VGG-16 [39] network to automatically detect COVID-19. Also, [48] applied a pretrained DenseNet201 [46] model on chest CT images to distinguish COVID-19 from non-COVID-19.

In [49], deep learning models and chest CT images differentiate coronavirus pneumonia from influenza pneumonia. This study was performed on CT images collected from various hospitals in China. Their studies have proven the effectiveness of CT images in diagnosing COVID-19. DeepPneumonia [50] was designed to classify COVID-19, bacterial pneumonia, and healthy cases based on CT images. Their proposed model achieved an accuracy of 86 : 5% for differentiating bacterial pneumonia and COVID-19 and 94% for distinguishing COVID-19 and healthy cases.

In [51], a new method called CONVNet based on the 3D deep learning framework for COVID-19 identification has been developed. This method can extract three-dimensional and two-dimensional representations. This method used ResNet [44] architecture. In [52], a deep transfer learning algorithm was introduced that used X-ray and CT scan images to accelerate the detection of COVID-19 cases. In [53], an attention-based deep learning model using the attention module with VGG-16 has been proposed. This method captures the spatial relationship between the ROIs in chest X-ray images. In [54], a new method based on BoVW (Bag of Visual Words) features has been proposed, which by removing the feature map normalization step and adding the deep features normalization step on the raw feature maps helps preserve the semantics of each feature map that may have important clues to differentiate COVID-19 from pneumonia.

### 2.3. Methods Based on Handcrafted Feature Extraction

Some COVID-19 detection methods used handcrafted feature extraction approaches. In [55], first, different texture features are extracted from the images by popular texture descriptors, and then, these texture features are combined with the extracted features from the pretrained Inception-v3 [56] model. In [57], a method for classifying the positive and negative cases of COVID-19 based on CT scan images was proposed. Different texture features were extracted from CT images using the Gabor filter, and then, the SVM method was used to classify these images. In [58], to reduce intensity variations between CT slices, a preprocessing step was applied on CT slices. Then, a long short-term memory (LSTM) classifier was used to discriminate between COVID-19, pneumonia, and healthy cases.

Other related methods based on the combination of feature extraction approaches and deep learning models are introduced in [59].

Most of the mentioned methods are highly dependent on the image domain of datasets on which they were trained. If the test set is from the same domain of the training set, the model performance will be acceptable. However, when the domain of the evaluation dataset is different, model performance is significantly reduced. However, in real-world applications, the domain of the inference image is not always the same as the training set. In other words, unseen data are often independent of the training set, so the results would not be reliable.

## 3. Proposed Approach: ADA-COVID

To overcome the mentioned problems in Section 1, we use the domain adaptation technique during model training. Using this technique during the training process, the generated representations do not depend on the domain of a particular dataset. Also, we use the triplet loss function for the training phase. Using this loss function, the distance between pairs of samples with similar classes in the embedded space is less than samples with different classes. Therefore, the extracted representations from the ADA-COVID model are very discriminative and domain invariant.

### 3.1. Overview

Figure 1 shows a general overview of the proposed method. As shown in this figure, different input domains are used in the COVID-19 detection process. The aim is to bring the statistical distribution of these domains closer together in the embedded space. The proposed method uses two different input domains named source and target. The source dataset is used to train the network, and the target dataset is applied for better generalizability of the network on new datasets. The next step is preprocessing, which includes decoding and resize, normalization, and augmentation. The output images from the preprocessing stage are entered into the ADA-COVID architecture. ADA-COVID consists of three modules as follows—(1) domain-invariant feature extractor: this module is responsible for extracting features, (2) classifier: this module is responsible for classifying data into two groups: COVID-19 and non-COVID-19, and (3) discriminator: this module is responsible for distinguishing and differentiating source data from target data.

The main aim of the proposed method is to generate similar representations for images belonging to two different domains. This model can perform the correct classification regardless of the specific features of each input distribution. Therefore, the model's generalizability increases, and it has the best performance for images belonging to different input domains.

The preprocessing step is introduced in Section 3.2, and the proposed ADA-COVID framework is described in Section 3.3.

### 3.2. Preprocessing

Preprocessing stage is performed to prepare data for training and evaluation of the model. The following paragraphs describe the different steps carried out in this regard.

#### 3.2.1. Decode and Resize

CT scan images are saved in DICOM file format, the widely used format in medical imaging. We need to convert DICOM format images to standard image formats such as JPG or PNG to work with such images. In the proposed method, we convert the images to grayscale PNG format.

In deep neural networks, input images are often resized to maintain compatibility with the network architecture and reduce computations [60]. The proposed method uses the pretrained ResNet50 architecture as a feature extractor with an input size of 224 × 224. Therefore, all images are resized into 224 × 224 pixels for training, validation, and testing.

#### 3.2.2. Normalization

To reduce the effect of intensity variations between CT slices, we normalize the data through (1) in the range [0, 1].

(1) $$\begin{array}{c} Z_{i}=\frac{X_{i}-\mu }{\sigma +\varepsilon }, \end{array}$$

where *x*_*i*_ represents the *i*-th image in the train set, and *μ* and *σ* represent the pixel level mean and standard deviation for all images in the train set, respectively. *ε*=1*e* − 10 is an insignificant value to prevent zero division, *i* is the index of each training sample, and *Z*_*i*_ is the normalized version of *X*_*i*_.

#### 3.2.3. Data Augmentation

Data augmentation means increasing the number of training samples by transforming images without losing semantic information. We use five transformations that are randomly applied to samples of the training set. These transformations are selected so that they do not lead to different interpretations by radiologists. The details of these transformations are summarized in Table 1.  Figure 2 shows some images after the preprocessing is applied.

### 3.3. ADA-COVID Framework

As shown in Figure 1, the ADA-COVID framework consists of three main modules: domain-invariant feature extractor, classifier, and discriminator. The following paragraphs describe these modules in detail. Also, the training procedure is provided in this section.

#### 3.3.1. Domain-Invariant Feature Extractor

This module is applied for extracting image features. Common CNN models such as VGG16 and ResNet are often used to extract features from images. These models require many training data to generate better representations. However, in the COVID-19 detection task, the size of the available datasets for network training is very small. Using transfer learning techniques is a practical solution to overcome this limitation. Transfer learning is a well-known representation learning technique in which the models trained on large image datasets (such as ImageNet [61]) are used to initialize the models for tasks for which the dataset is small. There are two general approaches to use transfer learning from pretrained models: feature extraction and fine-tuning [62]. In the first approach, only the weights of some newly added layers (classification layers) are optimized during training, while in the second approach, all the weights (or part of the weights) are optimized for the new task. In the proposed framework, we use the fine-tuning approach.

In the proposed framework, we use the pretrained ResNet50 [44] convolutional model trained on the ImageNet dataset. The ResNet50 has been selected after testing the most common pretrained CNN models. This architecture is smaller than other ResNet-based models (such as ResNet101 [44] and ResNet152 [44]) and has fewer parameters. Therefore, network training time is less than other models. An overview of the ResNet50 model is shown in Figure 3.

#### 3.3.2. Discriminator and Classifier

As described in Section 3.1, different input domains (source and target datasets) are used in the COVID-19 detection process. The discriminator module is responsible for differentiating source data from target data, and the classifier module is responsible for classifying data into two groups: COVID-19 and non-COVID-19.  Figure 4 illustrates an overview graphical representation of the model using the adversarial training approach in a multisource transfer learning setting. The classifier and discriminator utilize the features extracted by the feature extractor module at the same time to predict the class label and the domain from which the data came. The output predictor (classifier) and the domain classifier (discriminator) are trained classically by backpropagating their respective losses. When it reaches the feature extractor module, the gradient reversal layer reverses (multiplies by) (1) the domain classifier's loss. As a result, while the feature extractor learns a feature representation that is beneficial for output prediction, it also learns a feature representation that is indiscriminate of the domain from which the data come, promoting a more generalized one. The goal of learning representations using this joint architecture is to (1) generate representations that are indistinguishable from each other; (2) increase the model's generalizability; (3) learn representations that are based on essential features that are independent of the specific domain and dataset; and (4) distinguish COVID cases from non-COVID-19 cases with high accuracy.

The architecture of the discriminator and classifier modules is almost the same. In the discriminator module, we pass the extracted features into two consecutive blocks consisting of dense, batch normalization, ReLU, and dropout layers. On top of the discriminator module, we use the sigmoid function. The output of this function indicates the probability of assigning each sample to the source or target class. In the classifier module, in addition to two consecutive blocks consisting of dense, batch normalization, ReLU, and dropout layers, an embedding layer is added on top of the classifier module. This embedding layer is dense and has 64 neurons.

After training the network and learning the appropriate embedding, in the test phase, a dense layer with two neurons and a softmax activation function is added on top of the classifier module so that the network can be used independently as a classifier. Also, the discriminator module is no longer needed in the test phase, so this module is removed in the final application.

#### 3.3.3. Loss Function

Inspired by [63], we use two losses simultaneously in the network training process to increase the generalizability and transferability of the model. (2) represents the loss of the proposed method. This loss is a combination of a classifier loss (ℒ_*y*_) and a discriminator loss (ℒ_*d*_). *λ*_*d*_ and *λ*_*y*_ are the coefficients given to the discriminator and classifier losses, respectively. These coefficients are used to find the optimal balance between variance and bias for better generalizability of the model.

(2) $$\begin{array}{c} ℒ=\lambda_{y}{ℒ}_{y}+\;\lambda_{d}{ℒ}_{d}. \end{array}$$

We use the triplet loss function to calculate the classifier output loss (ℒ_*y*_) and the crossentropy loss function to calculate the discriminator domain loss (ℒ_*d*_).

Triplet loss was first introduced in FaceNet [64]. The idea is that pairs of samples in a class should have similar representations, and pairs of samples in different classes should have different representations in the embedded space. In triplet loss, a positive sample and a negative sample are selected for each sample (anchor). The positive sample is selected from the same class of the anchor sample, and the negative sample is selected from the opposite class of the anchor sample. Positive and negative samples are selected in each batch, and the loss function is calculated by (3).

(3) $$\begin{array}{c} {ℒ}_{y}=\text{Max}\left({\left\|f_{\theta }\left(A\right)-f_{\theta }\left(P\right)\right\|}^{2}-{\left\|f_{\theta }\left(A\right)-f_{\theta }\left(N\right)\right\|}^{2}+\alpha ,0\right), \end{array}$$

where, in (3), the function *f*_*θ*_ represents the data in embedded space and *θ* are parameters that must be learned. Thus, *f*_*θ*_(*A*), *f*_*θ*_(*P*), and *f*_*θ*_(*N*) represent embedded representations for the anchor, positive, and negative samples, respectively.  ‖‖^2^ represents the Euclidean distance, and *α* is a margin used to ensure that the model does not make the embeddings *f*_*θ*_(*A*), *f*_*θ*_(*P*),  and *f*_*θ*_(*N*) equal to each other to trivially satisfy the equation.

Due to the many inherent and structural similarities in medical images, the use of this loss function can be helpful to better differentiate data from two different classes in our task. The brilliant results of using this function in the present application reinforce the validity of this hypothesis.

We use the crossentropy loss function to calculate the discriminator domain loss (ℒ_*d*_). The crossentropy loss function is calculated by (4). In this equation, *y* represents the actual class, and $\hat{y}$ represents the model output prediction.

(4) $$\begin{array}{c} {ℒ}_{d}=-y\text{ log}\left(\hat{y}\right). \end{array}$$

## 4. Experiments

In this section, the performance of the ADA-COVID model is evaluated. The results are compared with the following groups of methods:

1. Methods that have developed customized network, such as COVID CT-Net [30], contrastive learning [35], Amyar et al. [13], Javaheri [36], xDNN [17], Wang et al. [65], Dadario et al. [66], Wu et al. [67], Liu [68], Singh et al. [69], He et al. [11], Zheng et al. [70], and Song et al. [50]
2. Methods that use pretrained networks and transfer learning to detect COVID-19, such as DenseNet201-based [48], modified VGG19 [52], ResNet-101-based [71], DenseNet-169-based [11], decision function [72], Chen et al. [29], Cifci [73], Jin et al. [74], Yousefzadeh et al. [75], DenseNet-169-based [76], and Wang et al. [77]
3. Methods that use handcrafted feature extraction approaches and conventional classifiers, such as Hasan et al. [58], Farid et al. [78], Xu et al. [79], Elghamrawy [80], and DenseNet-121 + SVM [4]

Parameter batch size and the maximum number of iterations are typical in the implemented methods, which are set to 32 and 2 × 10^4^, respectively. The learning rate in the ADA-COVID framework is set to 10^−2^ (in the ADA-COVID framework, Adam optimizer is used). In the proposed algorithm, the required parameters are set as follows: *λ*_*y*_=4, and *λ*_*d*_=1. Due to the small number of images, overfitting may occur. To solve this problem, dropout has been used along with the data augmentation technique. The dropout rate is set to 0.5. Also, the k-fold crossvalidation technique, considering *k* = 5, is used in the ADA-COVID framework. The experiments are conducted using the Keras framework on a computer with Intel (R) Core (TM) i7-7700K, 16 GB RAM, Nvidia GTX 1080 GPU.

To maximize the reliability of the proposed model, several slides of a patient's CT scan images are given to the network, and the average results are reported. In contrast, most of the compared methods reported the best results among different slides of a patient's CT scan images.

### 4.1. Dataset

To train and evaluate the model's performance and compare it with other methods, we use the SARS-CoV-2 CT scan dataset [17] as the source dataset and the COVID19-CT dataset [11] as the target dataset. The details of datasets are summarized in Table 2. 80% of the dataset is selected as a training set, and 20% of the dataset is selected as a test set.

### 4.2. Performance Metrics

The following five metrics are used to measure the performance in the experiments.

*Accuracy* is the number of correct predictions divided by the total number of samples [81]. This metric is calculated as follows.

(5) $$\begin{array}{c} \text{Accuracy}=\frac{TN+TP}{TN+TP+FN+FP}. \end{array}$$

*Precision* is the ratio of correct positive predictions to the number of positive results predicted. This metric is calculated as follows.

(6) $$\begin{array}{c} \text{Precision}=\;\frac{TP}{Tp+FP}. \end{array}$$

*Recall* is the ratio of the number of correct positive predictions to the number of all relevant samples. This metric is calculated follows.

(7) $$\begin{array}{c} \text{Recall }=\frac{TP}{TP+FN}. \end{array}$$

*F*_*1*_ *score* is the harmonic mean between precision and recall [82, 83]. This metric is calculated as follows.

(8) $$\begin{array}{c} {\text{F}}_{1}=2\times \frac{\text{Recall}\times \text{Precision}}{\text{Recall}+\text{Precision}}. \end{array}$$

*Specificity* rate corresponds to the proportion of negative samples that are correctly considered negative with respect to all negative samples. This metric is calculated by (9).

(9) $$\begin{array}{c} \text{Specificity}=\frac{TN}{TN+FP}. \end{array}$$

In equations (5) to (9), TP, FP, TN, and FN represent true positive, false positive, true negative, and false negative, respectively.

In our experiments, these metrics are expressed as a percentage. A high percentage indicates a better performance.

### 4.3. Experiment 1: Evaluation on the Source Dataset

This section compares the proposed approach's performance with the state-of-the-art methods on the source dataset, shown in Table 3. The results of other methods have been quoted directly from the relevant publications. Also, for the proposed method, the confusion matrix of evaluation on the test set of the source dataset is illustrated in Figure 5. From Table 3 and Figure 5, it is evident that ADA-COVID performs better than the other methods. It performs the best overall performance for all evaluation metrics. The average accuracy, precision, recall, and F1 metrics of ADA-COVID are 99.9%, 99.9%, 99.8%, and 99.9%, respectively. Recall 99.8% indicates that, on average, only one COVID-19 image is incorrectly predicted as non-COVID-19. Also, the proposed model correctly diagnoses all non-COVID-19 cases with only one false positive. After ADA-COVID, the EfficientNetB0, xDNN, DenseNet201-based, and ShuffleNet methods have relatively good performance, respectively. In EfficientNetB0 architecture, on average, two COVID-19 images are incorrectly predicted as non-COVID-19.

The visual evaluation results of ADA-COVID on 25 random samples from the test dataset are shown in Figure 6. Due to the model's high precision, there was no unsuccessful sample prediction in random results to examine the model's possible weaknesses.

### 4.4. Experiment 2: Evaluation on the Target Dataset

In this section, we evaluate the performance of the proposed approach on the target dataset once without training and once with training. In the first case, the model is trained on the source dataset and evaluated on the target dataset. In the second case, the proposed model is trained and evaluated independently on the target dataset. In other words, the second dataset input part and discriminator module are not considered in the second case, and the network is trained and evaluated on the target dataset. The performance of the different methods and models is shown in Table 4. The results of other methods have been quoted directly from the relevant publications. The compared methods are trained and evaluated on the target dataset.

As shown in Table 4, ADA-COVID with training on the target dataset has the best performance. The average accuracy, recall, specificity, and F1 metrics are 95.8%, 94.9%, 96%, and 95.2%, respectively. Also, after ADA-COVID with training, the ADA-COVID without training mode has the best performance. The average accuracy, recall, specificity, and F1 metrics are 92.5%, 93.5%, 94.2%, and 93%, respectively. In without training mode, the average recall of 93.5% indicates that, on average, eight images of COVID-19 are incorrectly predicted as non-COVID-19. Also, the average specificity of 94.2 indicates that all non-COVID-19 cases are detected with only seven false-positive samples. In training mode, the average recall of 94.9% indicates that, on average, 6 COVID-19 images are incorrectly predicted as non-COVID-19. Also, the average of specificity 96% indicates that it detects all cases of non-COVID-19 with only five false-positive samples.

In ADA-COVID without training mode, although the proposed approach is not trained on the target dataset, it has better results than other compared methods. This indicates that the proposed method has significantly increased generalizability, independent of the source dataset.

After ADA-COVID with and without training modes, the ResNet-50, ResNeXt-101, and ResNeXt-50 architectures have relatively good performance. In these architectures, the average recall of 92.16% indicates that, on average, more than 12 COVID-19 images are incorrectly predicted as non-COVID-19. Also, the average specificity of 90.2% indicates that all non-COVID-19 cases are detected with 15 false-positive samples. Among the reported results, AlexNet has the worst performance.

### 4.5. Experiment 3: Crossdataset Evaluation

To investigate the effect of the domain adaptation used in our approach on the final results, we evaluate the proposed approach's performance once with domain adaptation and once without domain adaptation. Also, we train the model once on the source dataset and evaluate it on the target dataset, and once on the target dataset and evaluate it on the source dataset. We compare the proposed method with the method proposed by Silva et al. [22] as the baseline. As shown in Table 5, the proposed method performs better than the reverse case when trained on the source dataset and evaluated on the target dataset. The reason for this is that the size of the target dataset is much smaller than the size of the source dataset. Also, the data collected in this dataset are from different sources, in different contrasts and with different visual features. Therefore, it is not a suitable dataset for the model training. Comparison of the proposed method with baseline [22] shows that the proposed method has improved the results by an average of 30%.

As shown in Table 5, the proposed approach performs better with the domain adaptation technique than without domain adaptation mode. Using the domain adaptation technique, the proposed approach results are improved by an average of 44.10%. Therefore, it can be concluded that better representations are generated by using the domain adaptation technique. As a result, the quality of the diagnoses is better, specifically for the unseen new samples.

### 4.6. Experiment 4: ADA-COVID vs. Pretrained Models

We evaluate the proposed method with methods in which the models are already pr-trained on the ImageNet dataset. As shown in Table 6, the results show that the proposed algorithm has a higher performance than other successful methods in this field. The critical point is that the proposed method is trained on the small SARS-CoV-2 CT scan dataset, while the other methods are often trained on a large dataset. Therefore, apart from the qualitative contributions and the proposed innovations that offer a low-cost and practical solution to overcome the shortcut learning problem [26], the proposed method achieves significant improvements using only a few sets of training samples without suffering from overfitting problem.

The method presented by Ardakani et al. [84] has almost higher performance than ADA-COVID in terms of recall metric; however, it suffers from low reliability. In other words, network performance decreases dramatically in the face of unseen data.

### 4.7. Experiment 5: ADA-COVID vs. Customized Models

This section compares the proposed method with methods that have developed customized architectures specifically to detect COVID-19. In these methods, transfer learning is not used, and the network is trained from scratch.

Table 7 shows the results for ADA-COVID and other compared approaches. As shown in this table, the ADA-COVID method, for all metrics, has the best results. After ADA-COVID, Elghamrawy and Hassanien [80] have the second-best results. Moreover, Hasan et al. [58] have relatively good performance. Wang et al. [77] have the worst performance among the reported results.

## 5. Conclusion

Rapid diagnosis of COVID-19 with high reliability is vital in the early stages of the infection. Using the transfer learning technique, this paper proposed an adversarial deep domain adaptation-based approach (ADA-COVID) for COVID-19 diagnosis from lung CT scan images. Previous studies suffer from shortcut learning when the model is trained using limited train data; furthermore, the state-of-the-art approaches fail to generalize for new samples, achieving poor performance or behaving similar to random predictors. Thanks to the proposed domain adaptation between the source and unseen target samples, ADA-COVID guarantees that the generated representations do not depend on the domain of a specific dataset. In addition, since medical images have a high structural resemblance compared to other image data in machine vision tasks, we utilized the triplet loss function for training the proposed model to achieve improved discrimination between positive and negative samples. Finally, the proposed approach can be easily extended for similar applications which utilize medical imaging such as radiography. ADA-COVID's performance was tested and compared to many state-of-the-art approaches. The results demonstrated that ADA-COVID achieves significant classification improvements, up to 60%, compared to the best results of competitors, even without directly training on the same dataset.

## Figures and Tables

**Figure 1:** Diagram of the proposed approach.

**Figure 2:** Preprocessed samples. (a) COVID-19 and (b) non-COVID-19.

**Figure 3:** Domain-invariant CNN encoder based on ResNet-50 architecture.

**Figure 4:** General representation of a deep model trained with the adversarial training methodology in the multisource transfer learning setting.

**Figure 5:** Confusion matrix of evaluation on the test set of the source dataset.

**Figure 6:** Performance evaluation on 25 random samples from the test set. “I” is the image index, “P” is the predicted value, and “L” is the ground truth label.

**Table 1:** Transformations.

Augmentation	Range/type
Brightness	[−10%, +10%]
Contrast	[−10%, +10%]
Rotation	[−20°, +20°]
JPEG noise	[50, 100]
Flip	Horizontal

**Table 2:** Characteristics of the utilized datasets.

Datasets	No. of samples	No. of COVID-19 samples	No. of non-COVID-19 samples	Image size
SARS-CoV-2 CT scan (source dataset)	2482	1252	1230	119 × 104 416 × 512

COVID-19 CT (target dataset)	746	349	397	124 × 153 1485 × 1853

**Table 3:** Performance comparison of different models for detecting COVID-19 on the source dataset (the best rates are bold-faced)

Model/method	Evaluation metrics			
	Accuracy	Precision	Recall	F_1_
AdaBoost	95.1	93.6	96.7	95.1
AlexNet	93.7	94.9	92.2	93.6
Decision tree	79.4	76.8	83.1	79.8
EfficientNetB0	98.9	99.1	98.9	99.0
GoogleNet	91.7	90.2	93.5	91.8
ResNet50	94.9	93.0	97.1	95.0
ResNet50V2	94.2	92.8	96.7	94.1
ShuffleNet	97.5	96.1	99.0	97.5
SqueezeNet	95.1	94.2	96.2	95.2
VGG-16	94.9	94.0	95.4	94.9
Xception	98.8	99.0	98.6	98.8

Contrastive learning [35]	90.8	95.7	85.8	90.8
COVID CT-Net [30]	90.7	88.5	85.0	90.0
DenseNet201-based [48]	96.2	96.2	96.2	96.2
Modified VGG19 [52]	95.0	95.3	94.0	94.3
xDNN [17]	97.3	99.1	95.5	97.3

**ADA-COVID**	**99.9**	**99.9**	**99.8**	**99.9**

**Table 4:** Performance comparison of different models for detecting COVID-19 on the target dataset.

Model/Method	Evaluation metrics			
	Accuracy	Recall	Specificity	F_1_
AlexNet	74.5	70.4	79.0	75.0
DenseNet-121	88.9	88.8	88.9	88.2
DenseNet-169	91.2	93.3	88.9	90.8
DenseNet-201	91.7	88.6	94.1	91.9
GoogleNet	78.9	75.9	82.3	79.0
Inception-ResNet-v2	86.3	88.1	84.2	87.0
Inception-v3	89.4	90.0	88.9	88.8
MobileNet-v2	87.2	93.2	77.6	89.0
NasNet-large	85.2	79.3	91.9	84.0
NasNet-Mobile	83.4	84.8	81.9	85.0
ResNet-101	89.7	82.2	89.2	89.0
ResNet-18	90.1	89.4	90.9	91.0
ResNet-50	90.8	90.0	91.0	90.1
ResNeXt-101	90.9	93.1	88.9	90.6
ResNeXt-50	90.6	93.4	88.2	90.3
ShuffleNet	86.1	83.5	89.0	86.0
SqueezeNet	78.5	86.5	63.8	82.0
VGG-16	78.5	74.6	82.8	76.0
VGG-19	83.2	90.7	74.7	85.0
Xception	85.6	88.3	80.6	87.7

Contrastive learning [35]	78.6	78.0	77.0	78.8
Decision function [72]	88.3	87.0	87.9	86.7
DenseNet-121 + SVM [4]	85.9	84.9	86.8	86.2
DenseNet-169-based [11]	83.0	84.8	85.5	81.0
DenseNet-169-based [76]	87.7	85.6	86.9	87.8
ResNet-101-based [71]	80.3	85.7	86.0	81.8

**ADA-COVID (without training)**	**92.5**	**93.5**	**94.2**	**93.0**
**ADA-COVID (with training)**	**95.8**	**94.9**	**96.0**	**95.2**

**Table 5:** Crossdataset evaluation results.

Method	Training dataset	Test dataset	Evaluation metrics		
			Accuracy	Recall	Precision
*Baseline*	Source	Target (train set)	59.12	64.14	54.95
	Source	Target (test set)	56.16	53.06	54.74
	Source	Target (all data)	58.31	61.03	54.90
	Target	Source	45.25	54.39	46.36

*ADA-COVID* (without domain adaptation)	Source	Target (train set)	64.28	65.10	64.12
	Source	Target (test set)	62.05	63.30	62.00
	Source	Target (all data)	65.37	66.80	65.22
	Target	Source	57.00	59.41	56.88

*ADA-COVID* (with domain adaptation)	Source	Target (train set)	91.04	92.70	92.11
	Source	Target (test set)	90.88	91.00	91.90
	Source	Target (all data)	**92.49**	**93.53**	**92.47**
	Target	Source	83.07	87.51	84.26

**Table 6:** ADA-COVID vs. pretrained models.

Reference	Data sources	No. of samples	Model	Performance
Ardakani et al. [84]	Real-time data from the hospital environment.	Total: 1,020 COVID-19 : 510 Non-COVID-19 : 510	AlexNet, VGG-16, VGG-19,…	Accuracy: 99.51 Recall: **100** Specificity: 99.02
Chen et al. [29]	Renmin Hospital of Wuhan University.	Total: 35,355	UNet++	Accuracy: 98.85 Recall: 94.34 Specificity: 99.16
Cifci [73]	Kaggle benchmark dataset [85]	Total: 5,800	AlexNet, Inception-V4	Accuracy: 94.74 Recall: 87.37 Specificity: 87.45
Javaheri et al. [36]	Five medical centers in Iran, SPIE-AAPM-NCI [86], LUNGx [87]	Total: 89,145 COVID-19 : 32,230 Non-COVID-19 : 56,915	BCDU-Net (U-Net)	Accuracy: 91.66 Recall: 87.5 Specificity: 94
Jin et al. [74]	Wuhan Union Hospital, LIDC-IDRI [88], ILD-HUG [89]	Total: 1,881 COVID-19 : 496 Non-COVID-19 : 1,385	ResNet152	Accuracy: 94.98 Recall: 94.06 Specificity: 95.47 F1: 92.78
Jin et al. [65]	Five different hospitals of China.	Total: 1,391 COVID-19 : 850 Non-COVID-19 : 541	DPN-92, Inception-v3, ResNet-50	Recall: 97.04 Specificity: 92.2
Li et al. [66]	Multiple hospitals environment.	Total: 4,536 COVID-19 : 1,296 Non-COVID-19 : 1,325	ResNet50	Recall: 90 Specificity: 96
Wu et al. [67]	China Medical University, Beijing Youan Hospital.	Total: 495 COVID-19 : 368 Non-COVID-19 : 127	ResNet50	Accuracy: 76 Recall: 81.1 Specificity: 61.5
Xu et al. [79]	Zhejiang University, Hospital of Wenzhou, Hospital of Wenling.	Total: 618 COVID-19 : 219 Non-COVID-19 : 399	ResNet18	Accuracy: 86.7 Recall: 81.5 F1: 81.1
Yousefzadeh et al. [75]	Real-time data from the hospital environment.	Total: 2,124 COVID-19 : 706 Non-COVID-19 : 1,418	DenseNet, ResNet, Xception, EcientNetB0	Accuracy: 96.4 Recall: 92.4 Specificity: 98.3 F1: 95.3

**ADA-COVID**	SARS-CoV-2 CT scan dataset	Total: 2,482 COVID-19 : 1,252 Non-COVID-19 : 1,229	ResNet50	Accuracy: **99.96** Recall: 99.80 Specificity: **99.80** F1: **99.90**

**Table 7:** ADA-COVID vs. customized models.

Reference	Data sources	No. of samples	Model	Performance
Amyar et al. [13]	COVID CT [16], COVID-19 CT segmentation dataset [90], Henri Becquerel Center	Total: 1,044 COVID-19 : 449 Non-COVID-19 : 595	Encoder-decoder with multilayer perceptron	Accuracy: 86.0 Recall: 94.0 Specificity: 79.0
Elghamrawy and Hassanien. [80]	COVID-19 database [91], COVID CT [16]	Total: 583 COVID-19 : 432 Non-COVID-19 : 151	WOA-CNN	Accuracy: 96.40 Recall: 97.25 Precision: 97.3
Farid et al. [78]	Kaggle benchmark dataset [85]	Total: 102 COVID-19 : 51 Non-COVID-19 : 51	CNN	Accuracy: 94.11 Precision: 99.4 F1: 94.0
Hasan et al. [58]	COVID-19 [92], SPIE-AAPM-NCI lung nodule classification challenge dataset [86]	Total: 321 COVID-19 : 118 Non-COVID-19 : 203	QDE–DF	Accuracy: 99.68
He et al. [11]	COVID-19 database [91], COVID-19 [92], Eurorad [93], corona cases [94]	Total: 746 COVID-19 : 349 Non-COVID-19 : 397	CRNet	Accuracy: 86.0 F1: 85.0 AUC: 94.0
Liu et al. [68]	Ten designated COVID-19 hospitals in China	Total: 1,993 COVID-19 : 920 Non-COVID-19 : 1,073	Modified DenseNet-264	Accuracy: 94.3 Recall: 93.1 Specificity: 95.1
Singh et al. [69]	COVID-19 patient chest CT images [95]	Total: 150 COVID-19 : 75 Non-COVID-19 : 75	MODE-CNN	Accuracy: 93.25 Recall: 90.70 Specificity: 90.72
Wang et al. [77]	Xi'an Jiaotong University, Nanchang University, Xi'an Medical College	Total: 1,065 COVID-19 : 740 Non-COVID-19 : 325	Modified inception	Accuracy: 79.3 Recall: 83.0 Specificity: 67.0
Song et al. [50]	Hospital of Wuhan University, third affiliated hospital	Total: 1,990 COVID-19 : 777 Non-COVID-19 : 1,213	DRE-Net	Accuracy: 94.3 Recall: 93.0 Precision: 96.0
Zheng et al. [70]	Union Hospital, Tongji Medical College, Huazhong University of Science and Technology	Total: 630	DeCoVNet	Accuracy: 90.1 Recall: 90.7 Specificity: 91.1

**ADA-COVID**	SARS-CoV-2 CT scan dataset	Total: 2,482 COVID-19 : 1,252 Non-COVID-19 : 1,229	ResNet50	Accuracy: **99.96** Recall: 99.80 Specificity: **99.80** F1: **99.90**

## Data Availability

Previously reported image data were used to support this study and are available at doi.org/10.1101/2020.04.24.20078584 and https://doi.org/10.1101/2020.04.13.20063941. These prior studies (and datasets) are cited at relevant places within the text as references [11, 17].
